The article "Root foraging of birch and larch in heterogeneous soil nutrient patches under water deficit" was retracted in 2024. Reasons: concerns about the peer review; concerns about the citations; concerns about a third party's involvement.

# Root foraging of birch and larch in heterogeneous soil nutrient patches under water deficit

**DOI:** 10.1371/journal.pone.0255848

**Published:** 2021-08-10

**Authors:** Long Tan, Ruifeng Fan, Huifeng Sun, Shenglei Guo

**Affiliations:** 1 College of Pharmacy, Heilongjiang University of Chinese Medicine, Harbin, China; 2 Harbin Gloria Pharmaceuticals Ltd., Harbin, China; Shandong University, CHINA

## Abstract

Water and nutrient are two critical factors that limit plant growth to spatial-temporal extents. Tree root foraging behavior has not received adequate attention in heterogeneous soil environments in temperate forest under drought pressure. In this study, birch (*Betula platyphylla*) and larch (*Larix olgensis*) seedlings were raised in pots in a split-root system with artificially heterogeneous soil environments to study the root foraging response to drought. Potted space was split into two halves where substrates were mixed with fertilizers in 67.5 mg nitrogen (N) plant^-1^ (N-P_2_O_5_-K_2_O, 14-13-13) to both halves as to create a homogeneous condition. Otherwise, a rate of 135 mg N plant^-1^ of fertilizers was delivered to a random half to create a heterogeneous condition. Half of seedlings were fully sub-irrigated every three days with the other half received the drought treatment by being watered every six days. Both birch and larch seedlings showed greater net shoot growth and biomass increment in well-watered condition, while root morphology was promoted by drought. Both species placed more fine roots with higher root N concentration in nutrient-enriched patches. In the heterogeneous pattern, birch showed a higher foraging precision assessed by biomass and greater foraging plasticity assessed in morphology and physiology. In contrast, larch seedlings had higher root N concentration in the well-watered condition. Neither species showed a significant response of N utilization to the heterogeneous pattern, but both used more N when water supply was improved. Overall, birch is better at acclimating to heterogeneous soil conditions, but its ability to seize N was lower than larch when drought was alleviated.

## Introduction

Widespread drought-induced tree mortality may be underestimated as a natural ecological process [1]. Exposure of forests to drought events in the current scenario of climate change has a close relation to tree mortality [2, 3]. Forests may become increasingly vulnerable to future droughts, even in regions that have rarely had issues of limited water [2]. An extreme drought event can continuously reduce growth of deep-rooted forest trees for as long as four years [4, 5]. Knowledge about tree response to drought is necessary to better understand the forest ecosystem response to warming climate.

As a major source for water and carbon exchanges between atmosphere and soils, tree roots are well equipped to withstand drought situations and maintain eco-physiological functions [6]. Tree roots are capable of responding to drought through a variety of strategies including belowground biomass adjustment, anatomical alteration, physiological acclimation, and morphological growth [6]. A drought event can stimulate tree roots to penetrate downwards and explore deeper soils by elongating the root axis and enlarging the diameter and surface area of the root system [7, 8]. More roots arranged in deeper soils can compensate for declining shallow roots in severe droughts [8] and avoid competition for water in topsoil [7]. Tree root systems can also increase the branching of lateral fine roots by continuously egressing new roots to arrange the belowground system and help increasing soil porosity [9]. Furthermore, strong variation of root response to drought exists among different tree species [10]. All these findings together suggest a potential promotion of fine root proliferation in drought for patchy soil micro-sites. However, there is little documentation about the foraging behavior of fine roots in heterogeneous soil environments under water deficit conditions.

Organic fractions in soils are established by the input of leaf litter, dead roots, animal corpses, and dead micro-organisms [11]. Uneven microbial activity decomposing these organic materials and the subsequent diffusion of released inorganic ions result in a heterogeneous soil environment with patches of various nutritional availabilities [12]. Patchy distribution of resources is the source of heterogeneous soil environment that drives root proliferation. Drought can modify composition of the soil bacterial community [13] and alter decomposition processes [14, 15]. Therefore, drought can further interrupt biogeochemistry and N cycling [15, 16] possibly affecting fine root foraging behavior. It is necessary to assess root foraging behavior in order to determine precise fine root response to heterogeneous soil patches under water deficit conditions.

Plant roots have the ability to proliferate in soils towards nutrient-enriched patches, i.e., the ‘foraging behavior’ [12, 17]. This is mainly achieved by elongating fine root axis and increasing the number of branching tips, as well as expanding fine root surface-area [12, 18–22]. Fine root foraging in heterogeneous patches can be evaluated by the parameters of ‘scale’ and ‘precision’. Root foraging scale determines the extent to which fine roots can be placed in nutrient enriched patches [23] which is related to species variation and growth rate [23–26]. Foraging scale determines root size and both are distributed depending on the pattern of heterogeneous soil resources. Root foraging precision is fine root difference in soil patches with contrasting nutritional enrichments [23, 26, 27]. Foraging precision can be taken as the ability of fine roots to be placed in nutrient-rich patches [28]. The combination of these parameters can contribute to a better understanding of tree root foraging in response to drought. The heterogeneous nutrient pattern may impact nutrient availability regarding uptake from root foraging. Therefore, N utilization may also be changed in heterogeneous soils compared to former studies where it was hypothesized that soils were homogeneous. Nitrogen utilization has been found to have a close relationship with the variation of N availability [29–32]. However, to our knowledge little has been documented about N utilization of trees with roots in heterogenous soil patches. Quantifying N utilization in drought will also create a deeper understanding of N acquirement efficiency when facing drought conditions.

Temperate forests in the Northern Hemisphere are expected to undergo future drought events with high frequency and increasing severity [33]. Birch and larch are two early successional timber species that are sensitive to climatic drought and are used as model plants to study tree response to water deficit [34–36]. Potted plants are commonly used in controlled experiments of studies that detected root foraging behavior in heterogeneous soil patches [11, 23, 25, 26, 37]. In this study, seedlings of white birch (*Betula platyphylla*) and Changbai larch (*Larix olgensis*) were cultured in pots where patches of substrates were fed by fertilizers to simulate heterogeneous soil environments. Some seedlings were cultured with water deficit by limiting irrigation while others were watered well. Regarding the similar response to soil heterogeneous condition across multiple herbaceous plant species [12, 23, 38], our objective was to assess fine root foraging behavior and N utilization in the two tree species. It was hypothesized that: (i) root foraging precision and plasticity will show the same response for both birch and larch, and (ii) root foraging behavior will be promoted by drought [7, 8].

## Materials and methods

### Study site and experimental conditions

This study was conducted in a growth chamber in the Laboratory of Combined Manipulation of Illumination and Fertility on Plant Growth (Zhilunpudao Agric. For. Sci. Ltd., Changchun, China). The laboratory was sealed to avoid ambient sunlight and wind. All illumination that was used for seedling culture was supplied by lighting panels that were embedded with light-emitting diodes (LEDs). Diodes emitting red (R), green (G), and blue (B) lights were embedded to a panel to irradiate the spectrum of 16.6/75/8.4 (R/G/B) wavelength. Electric current was controlled by a 140-W transformer. More details can be found in Wei et al. [39]. The photosynthetic photon flux rate (PPFD) for seedling growth was set in the range of 70–200 μmol m^-2^ s^-1^ which was successfully used for tree seedling culture [30, 40]. The spectrum was composed by PPFD ratios of 85% red, 5% green, and 10% blue lights, which contributed to standard wavelengths for tree seedling growth [30, 41]. Seedlings were cultured with an 18 h photoperiod from 06:00 a.m. to 24:00 p.m. [40, 41]. Temperature was maintained between 17.2/31.7°C (night/day). Relative humidity (RH) ranged in 15–61% under drought condition and in 77–93% with ordinary watering.

### Seedling material

Seeds of white birch (*Betula platyphylla*) and Changbai larch (*Larix olgensis*) were supplied by Harbin Gloria Pharmaceuticals Limited. This affiliation issued the authority for field permission to collect seeds. Seeds of both species were collected from four mother trees in a narrow geographical range to avoid the genetic-variation effect. Stratified seeds were sterilized using 5% potassium permanganate (w/w) soaked in water for 12 h and sown in acid-washed sand. Seeds were incubated in a chamber under the constant condition of 28°C temperature and 80% (RH). When germination was completed, seedlings were transplanted to purified peat substrate (Zhiluntuowei A&F Sci. Inc., Changchun, China) and treated by commercial fertilizers (N-P_2_O_5_-K_2_O, 20-20-20, Everris^TM^, Geldermalsen, The Netherlands). Fertilizer was delivered twice a week through eight applications to a total amount of 20 mg N plant^-1^ to support the basic growth from germinates to initial seedlings with full expansion of first leaves. During this period, seedlings were cultured under PPFD panels to receive PPFD of 70–73 μmol m^-2^ s^-1^ in a daily photoperiod of 18 h. For birch and larch seedlings, initial height was 11.37 cm and 5.76 cm while initial root-collar diameter (RCD) was 0.35 cm and 0.08 cm, respectively. Twenty seedlings of each species were divided into parts of shoot and root, which were both dried in an oven at 70°C for 72 h and prepared for further measurements.

### Experiment design and substrate manipulation

The experiment was conducted as a 2×2 factorial design arrangement with two water-condition regimes (drought-stressed vs. well-watered), and two nutritional enrichment patterns (heterogeneous vs. homogeneous). Forty-eight 0.45-L pots (top diameter × bottom diameter × height, 11.5 × 7.5 × 9.5) were arranged in six replicated blocks which were randomly placed after every watering to tanks. Eight pots assigned for eight combined treatments were placed in one plastic tray (length × width, 75 cm × 25 cm) as a block and six trays were assigned as six replicates of combined treatments (*n* = 6). Commercial substrates of mixed peat and perlite (3/1, v/v) (Mashiro-Dust^TM^, Zhiluntuowei Agric. For. Sci. Inc., Changchun, China) were fully soaked by distilled water and used to fill up pots to the height of 4 cm above the bottom. The substrate had mineral N of 164 mg kg^-1^, available P of 0.2 g kg^-1^, organic matter of 11%, pH of 4.8, and electrical conductivity of 1.2 μS cm^-1^ that can fully facilitate plant growth [42–44]. Potted substrates were divided into two halves by inserting a piece of plastic sheet vertically in the middle section of each pot at the height of 7.5 cm. Half of the pots (*n* = 24) were assigned as the treatment with homogenous nutritional patches. This was achieved by adding the same amount of 67.5 mg N of granules of controlled-release fertilizers (CRFs) (N-P_2_O_5_-K_2_O, 14-13-13, No.5 Osmocote^®^, The Scotts Co., Marysville, OH, USA) to both halves of the pot. The remaining pot spaces (*n* = 24) were assigned as the treatment with heterogeneous nutritional patches by adding 135 mg N to a random half of the pot through CRF granules with the other half receiving nothing. These manipulations of nutritional patch formation were adapted from Wei et al. [11]. The remaining space of each pot was filled by water-soaked substrate to the top. On one hand, data can be analyzed by two water deficit levels and two patterns (heterogeneous vs homogeneous); and on the other hand, data can also be analyzed by two water deficit levels combining three half-pot nutrient availabilities (low, medium, and rich levels). Roots of initial seedlings were cut to leave 30% of total length by rough visual estimation. Thereafter, seedlings were transplanted to the middle of the top surface of every pot at the density of one seedling per pot.

### Drought treatment

The well-watered treatment was achieved by watering pots to full capacity every three days [36]. In the drought treatment, water deficit was brought about by watering seedlings every six days [36]. The amount of water irrigated to seedlings under deficit condition was 70 ml per pot. In the past 110 years (1905–2010), the historical record of minimum precipitation that caused drought events in Northeast China was about 200 mm in two months during summer [45]. Therefore, the amount of water input to seedlings every six days was 20 mm. This arrangement equaled 70 ml in total with a hypothesis that all water was evenly input into a column with top diameter of 11.5 cm.

### Harvest and measurement

The experiment lasted for four months until both birch and larch seedlings started to show dehydration symptoms of yellow leaves and dieback of shoot tips (Fig 1). All seedlings were harvested in three steps. Firstly, seedlings were cut into shoot and root at the root collar on the surface of the substrate. The shoot was thereafter used for measurements of height and root-collar diameter (RCD; the diameter 1.5 cm above the cutting scar). Net shoot growth and biomass of final absolute values minus initial ones were used as the parameters for shoot. Secondly, roots were split into two halves by shearing from the top of the tap root along the plastic sheet in the substrate. This manipulation ensured that roots were harvested separately from each side of the two compartments. Finally, all roots were carefully excavated out of each half of the substrate minimizing loss of fine roots. Harvested roots were carefully rinsed in tap water to remove attached substrates at the surface, then they were washed with distilled water. Roots were scanned to generate a projected image at the resolution of 118.11 pixels cm^-1^ (HP Deskjet 1510 scanner, HP Inc., Palo Alto, CA, USA). Root images were analyzed by the WinRHIZO software (Regent Ltd., Alberta, Canada) to quantify fine root morphologies of length, surface area, and tip number. All harvested parts (shoot, left-patch roots, and right-patch roots), as well as the pre-sampled seedling parts prior to the experiment, were oven-dried at 70°C for 72 h and were all measured for dry weight. Dried samples were ground to pass a 60-mesh (0.25 mm) sieve [46]. Ground samples were digested in 5 mL of hydrogen peroxide-sulfuric acid, diluted to 50 mL, and determined for N concentration using the Kjeldahl method [30].

**Fig 1:** Performance of birch and larch seedlings cultured in heterogeneous and homogeneous nutrient environments in pots with drought and well-watered conditions.

### Parameter calculation

Root foraging precision was evaluated by the absolute difference of fine root parameters between halves of pot patches [11]:

FRMD=|finerootmassinleftpatch−finerootmassinrightpatch| (1)

FRLD=|finerootlengthinleftpatch−finerootlengthinrightpatch| (2)

FRSD=|finerootsurfaceareainleftpatch−finerootsurfaceareainrightpatch| (3)

FRND=|finerootNconcentrationinleftpatch−finerootNconcentrationinrightpatch| (4)

where FRMD, FRLD, FRSD, and FRND are fine root differences of mass, length, surface-area, and N concentration between two halves of pot patches, respectively. Fine root foraging plasticity was evaluated by N uptake per root unit [37]:

$$NUPL=\frac{{Root}_{N}}{{Root}_{L}}$$ (5)

$$NUPM=\frac{{Root}_{N}}{{Root}_{M}}$$ (6)

where NUPL and NUPM are N uptake per fine root length and per fine root mass, respectively. *Root*_*N*_ is fine root N concentration, *Root*_*L*_ is fine root length, *Root*_*M*_ is fine root mass. According to Wang et al. [37], NUPL and NUPM can be used for assessing morphological and physiological plasticity, respectively. The index of N utilization (NUI) was calculated by the model [29]:

$$NUI=\frac{{Mass}_{Whole}}{{Foliar}_{N}}$$ (7)

where *Mass*_*Whole*_ is whole-plant biomass, *Foliar*_*N*_ is foliar N concentration.

### Statistical analysis

Statistical analyses were undertaken using SAS software (ver. 9.4 64-bit, SAS Institute, Cary, NC, USA). Data were tested for the normal distribution of standardized residuals according to Shapiro-Wilk test using the general linear model (GLM) procedure. Data were transformed by the box-cox methodology using the TRANSREG Procedure when abnormal data were detected (S1 Table). In addition to the normality test, Levene’s test was employed for standardized residuals to confirm the equal group variances of transformed data using the HOVTEST procedure. Taking the two species (birch vs larch) as split sets of data sources, results were nested to each of the species and can be analyzed by two types of factorial models. Furthermore, split data nested to either species were tested by two-way analysis of variance (ANOVA) for above-ground and below-ground organs separately. For shoot organs, a two-way ANOVA was used to test the sources of variance of water condition (drought vs well-watered) and nutrient distribution pattern (heterogeneous vs homogeneous). For root organs, another two-way ANOVA was used to test effects from water condition and half-pot patchy nutrient availability (poor, medium, and rich). Factors of water condition and nutrient distribution pattern were also used to detect foraging precision, plasticity, and N utilization. When significant interactive effects were indicated by ANOVA, means were compared and arranged by one-way ANOVA with combined treatments across factors. Significant effect of ANOVA was compared and arranged by means according to Duncan test (*α* = 0.05).

## Results

### Shoot growth, biomass, and nitrogen allocation

Water condition had a significant main effect on net increment in height and RCD growth and biomass accumulation (Table 1). Compared to the drought treatment, the well-watered condition resulted in higher net growth in height, RCD, and shoot biomass by 366%, 51%, and 315%, respectively, in birch seedlings. In larch seedlings, the countering drought treatment resulted in 138%, 63%, and 166% for the increments of these three variables, respectively (Fig 2). In addition, the nutrient distribution pattern also had a significant main effect on net height growth in larch seedlings. Larch seedlings in the heterogeneous pattern had a net height growth of 8.51±5.05 cm (mean ± standard deviation, the same below) compared to those in the homogeneous pattern (4.69±4.50 mm) with an increase of 81%.

**Fig 2:** Net growth in height (A), root-collar diameter (RCD) (B), and biomass (C) in birch (*Betula Platyphylla*) and larch (*Larix olgensis*) seedlings subjected to drought vs well-watered conditions. Bars indicate standard deviations. Different letters indicate significant difference of raw transformed data (see S1 Table) according to Duncan test at 0.05 level. Lower case letters stand for differences for birch seedlings and capital letters for larch seedlings.

**Table 1:** *F* values from Analysis of variance (ANOVA) of nutrient distribution pattern (P), water condition (W), and their interaction (P × W) on growth, biomass, and nitrogen (N) concentration in shoots of birch (*Betula Platyphylla*) and larch (*Larix olgensis*) seedlings.

Variables	Birch			Larch		
	P	W	P × W	P	W	P × W
Seedling height	0.55	60.31*** ^1^	0.16	5.38*	10.75*	0.19
RCD ^1^	0.01	25.80***	1.25	4.13	16.32**	1.16
Shoot biomass	0.06	60.73***	0.02	3.11	8.82*	0.10
Shoot N concentration	5.14*	0.01	20.07**	6.36*	19.54**	9.34*

Note: Asterisks indicate significance.

*, *P*<0.05

**, *P*<0.01

***, *P*<0.001. RCD, root-collar diameter.

Factors of nutrient distribution pattern and water condition had an interactive effect on shoot N concentration (Table 1). In birch seedlings, shoot N concentration was higher under drought condition in the heterogeneous pattern compared to that under well-watered condition in the heterogeneous pattern or under drought condition in the homogeneous pattern (Fig 3A). In larch seedlings, the drought condition in the heterogeneous pattern resulted in a higher shoot N concentration than the other treatments combined.

**Fig 3:** Nitrogen (N) concentration in shoots of birch (*Betula Platyphylla*) and larch (*Larix olgensis*) seedlings subjected to drought vs well-watered conditions in heterogeneous or homogeneous nutrient patterns. Bars indicate standard deviations. Different letters indicate significant difference of raw transformed data (see S1 Table) according to Duncan test at 0.05 level. Lower case letters stand for differences for birch seedlings and capital letters for larch seedlings.

### Fine root morphology, biomass, and nitrogen uptake

Either factor of half-pot patchy nutrient availability or water condition had a main effect on fine root morphology, biomass, and N concentration (Table 2). Birch seedlings had lower levels in fine root length, surface-area, tip-number, and biomass for fine roots in half-pot patches with poor N availability compared to those in medium and rich availabilities (Fig 4A, 4C, 4E and 4G). In larch seedlings, the fine root variables of length, surface-area, tip-number, and biomass were always higher for fine roots in patches with rich N availability relative to those with low N availability. However, the difference of fine root variables between medium and the other two availabilities was not always significant. The well-watered condition resulted in higher fine root length, surface-area, tip-number, and biomass compared to those under the drought condition for both birch and larch seedlings (Fig 4B, 4D, 4F and 4H).

**Fig 4:** Fine root length (A, B), surface-area (C, D), tip-number (E, F), and biomass (G, H) in birch (*Betula Platyphylla*) and larch (*Larix olgensis*) seedlings subjected to heterogeneous or homogeneous nutrient patterns (left) or in drought vs well-watered conditions (right). Bars indicate standard deviations. Different letters indicate significant difference of raw transformed data (see S1 Table) according to Duncan test at 0.05 level. Lower case letters stand for differences for birch seedlings and capital letters for larch seedlings.

**Table 2:** *F* values from analysis of variance (ANOVA) of patchy nutrient availability (PA), water condition (W), and their interaction (PA × W) on morphology, biomass, and nitrogen (N) concentration in roots of birch (*Betula Platyphylla*) and larch (*Larix olgensis*) seedlings.

Variables	Birch			Larch		
	PA	W	PA × W	PA	W	PA × W
FR length	9.52**	20.34***	1.64	3.59*	4.48*	1.00
FR surface-area	12.67***	30.64***	1.79	5.51**	7.11*	0.65
FR tip-number	6.49*	61.77***	0.21	6.09*	15.08**	0.03
Root biomass	4.38*	31.01***	0.22	6.97*	14.52**	2.72
Root N concentration	6.83**	0.01	2.99	22.23***	20.38***	1.74

Note: FR, fine root. Asterisks indicate significance.

*, *P*<0.05

**, *P*<0.01

***, *P*<0.001.

Patchy nutrient availability had a main effect on root N concentration in birch and larch seedlings, and water condition also had a main effect on root N concentration in larch seedlings (Table 2). Root N concentration was higher in half-pot patches with rich availability compared to that in the other two types of patches both in birch and larch seedlings (Fig 5A). Water condition did not affect root N concentration for birch seedlings. Instead, water condition differentiated root N concentration in larch seedlings (Fig 5B). The well-watered condition increased root N concentration by 65% compared to the drought condition.

**Fig 5:** Nitrogen (N) concentration in roots of birch (*Betula Platyphylla*) and larch (*Larix olgensis*) seedlings subjected to heterogeneous or homogeneous nutrient patterns (top) or in drought vs well-watered conditions (bottom). Bars indicate standard deviations. Different letters indicate significant difference of raw transformed data (see S1 Table) according to Duncan test at 0.05 level. Lower case letters stand for differences for birch seedlings and capital letters for larch seedlings.

### Root foraging precision

Either nutrient distribution pattern or water condition did not have interactive effect on FRLD, FRSD, and FRND (Table 3). However, they had an interactive effect on FRMD (Fig 6). Birch seedlings in the heterogeneous pattern had a higher FRMD compared to those in the homogeneous pattern. Larch seedlings subjected to the drought condition in the heterogeneous pattern had the highest FRMD.

**Fig 6:** Fine root mass difference (FRMD) in birch (*Betula Platyphylla*) and larch (*Larix olgensis*) seedlings subjected to drought vs well-watered conditions in heterogeneous or homogeneous nutrient patterns. Bars indicate standard deviations. Different letters indicate significant difference of raw transformed data (see S1 Table) according to Duncan test at 0.05 level. Lower case letters stand for differences for birch seedlings and capital letters for larch seedlings.

**Table 3:** *F* values from analysis of variance (ANOVA) of nutrient distribution pattern (P), water condition (W), and their interaction (P × W) on variables assessing root foraging plasticity and nutrient utilization in birch (*Betula Platyphylla*) and larch (*Larix olgensis*) seedlings.

Variables	Birch			Larch		
	P	W	P × W	P	W	P × W
FRMD	20.79***	1.02	1.38	3.10	3.27	4.99*
FRLD	0.55	0.23	0.20	0.03	3.99	0.86
FRSD	3.41	6.26	6.06	1.93	3.11	1.77
FRND	0.90	0.65	3.15	3.11	0.27	1.99
NUPL	4.89*	15.62***	0.42	0.50	13.14***	0.05
NUPM	1.82	28.63***	1.00	0.05	33.50***	0.56
NUI	0.32	35.90***	3.62	3.18	12.43**	0.22

Note: FRMD, fine root mass difference; FRLD, fine root length difference; FRSD, fine root surface-area difference; FRND, fine root nitrogen concentration difference; NUPL, nitrogen uptake per root length; NUPM, nitrogen uptake per root mass; NUI, nutrient uptake index.

### Foraging plasticity and nutrient utilization

The factor of nutrient distribution pattern had a main effect on NUPL, but its effect on NUPM was not significant (Table 3). The heterogeneous pattern resulted in higher NUPL by 45% in birch seedlings compared to the homogeneous pattern (Fig 7A). Water condition had a significant main effect on NUPL and NUPM in both birch and larch seedlings (Table 3). Compared to the drought condition, the well-watered condition increased NUPL by 47% and 358% for birch and larch seedlings, respectively (Fig 7B). The well-watered condition also resulted in an increase of NUPM by 101% and 229% for birch and larch seedlings, respectively (Fig 7D). The factor of nutrient distribution pattern did not cause any effect on NUI in birch and larch seedlings (Fig 7E). Compared to the drought condition, the well-watered condition resulted in an increase of NUI by 114% and 148% for birch and larch seedlings, respectively (Fig 7F).

**Fig 7:** Nutrient uptake per fine root length (NUPL) and per fine root mass (NUPM) and N utilization index (NUI) in birch (*Betula Platyphylla*) and larch (*Larix olgensis*) seedlings subjected to heterogeneous vs homogeneous nutrient patterns in drought or well-watered conditions. Bars indicate standard deviations. Different letters indicate significant difference of raw transformed data (see S1 Table) according to Duncan test at 0.05 level. Lower case letters stand for differences for birch seedlings and capital letters for larch seedlings.

## Discussion

### Fine root placement in heterogeneous patterns

Fine root morphology (length, surface-area, and tip-number) and biomass generally showed an increasing trend with patchy nutrient availability both in birch and larch seedlings. This is the result of precise placement of fine roots in nutrient enriched patches by the two tree species. Our results fully concur with previous findings on crop and herbaceous plants [12, 17]. A study on subtropical tree species also showed the same response to drought [47]. Hence, the plasticity of fine root length was higher in the heterogeneous pattern compared to the homogeneous pattern. These results concur to those of Wei et al. [11] where *Taxus cuspidata* seedlings failed to increase fine root morphology in nutrient enriched patches. Slow growers need more time to forage nutrients in microsites and proliferate fine roots therein. However, our fine roots subjected to nutrient enriched patches generally had larger morphology and greater biomass than those in poor patches, while fine roots between medium and rich patches showed no difference. This can be explained by the limit of foraging precision because the two tree species we tested cannot recognize medium to high levels of nutrient availabilities to place their fine roots. Therefore, foraging precision did not show any response to patchy nutrient availability when assessed by fine root morphologies. The responsive foraging precision that was assessed by fine root biomass was not the result of foraging because the physiological plasticity of fine root placement was not different between contrasting patterns. Absence of physiological plasticity in fine roots was also reported on *Pinus taeda* trees [37]. Thus, we can accept our first hypothesis.

Drought promoted foraging precision in the heterogeneous pattern for both birch and larch seedlings. The response of fine root biomass difference to the heterogeneous pattern in our results agree with those found on ten co-occurring plants [23] and *Pinus massoniana* seedlings [21]. To our knowledge, we are the first to find the promotion of drought on root foraging precision. We surmise this was caused by enlarged foraging scale [23] because drought can modify the extent of scale for root growth rate [23–26]. The first explanation to support our conclusion was that drought can promote all variables concerning fine root morphology and biomass which suggests an increase of foraging scale. The proliferation of fine roots and egress of new roots together represent a general response to cope with water deficit stress [8, 9, 48]. Our conclusion can also be supported by theoretical evidence from other studies. For example, Rajaniemi and Reynolds [38] reported a close positive relationship between root foraging scale and precision assessed by root mass in eight herbaceous plants. However, it was also reported that fine root foraging precision showed null response to nutritional patches in *Podocarpus macrophyllus* seedlings despite a larger foraging scale in heterogeneous substrate [11]. In addition, the relationship between foraging scale and precision was also found to be a tradeoff in eight herbaceous plants [27]. These studies together demonstrate an unconfirmed relationship between foraging scale and precision. In contrast, drought reduced fine root foraging plasticity in both morphology and physiology. This further suggests that the proliferation of fine roots in drought spent a greater cost of biomass investment for morphology growth and N uptake. Nevertheless, we can accept our second hypothesis.

### Nutrient uptake and utilization

Nitrogen in shoots is a critical trait that supports shoot growth and biomass accumulation. The drought effect on shoot N concentration was dependent on the substrate N distribution pattern. In our study, the drought condition increased shoot N concentration in birch and larch seedlings in the heterogeneous pattern. When N supply was attained from patchy sources, fine root foraging precision was increased for larch seedlings, causing shoot N concentration increase by enhancing N uptake efficiency. However, N foraging precision was unchanged in drought-treated birch seedlings in the heterogeneous pattern. We surmise that the increase of shoot N concentration in birch seedlings resulted from drought stress on shoots as reduced growth and biomass. This conclusion can be partly supported by decreases in shoot growth and biomass in drought-treated seedlings despite no response to the interactive effects. Shoot biomass declined and subsequent N concentration increase was also found in other tree species [49, 50]. We cannot speculate that N uptake accounted for shoot N concentration decline in birch because root N concentration therein was not changed by drought. More trials are needed to test the potential response of shoot N status to interactive water condition and nutrient supply pattern.

In the homogeneous pattern, shoot N concentration was depressed by drought for birch seedlings, but drought did not impact shoot N concentration in larch seedlings. In addition, neither foraging plasticity nor N utilization in larch seedlings were impacted by the nutrient pattern. These results together suggest that the larch species tested in this study did not have the same level of expected foraging precision as birch in the homogeneous pattern. According to field studies, larch had a lower fine root growth rate and biomass allocation than birch [51, 52]. Therefore, we attribute the null response of root plasticity and foraging precision in larch seedlings to low root proliferation. The heterogeneous nutrient pattern also failed to impact shoot N concentration in *Zea mays* [17], which coincides with our results for larch seedlings. Neither birch nor larch seedlings showed impacts from drought in the homogeneous pattern on root N concentration, hence we cannot attribute the change of shoot N concentration to uptake.

Birch seedlings had higher foraging precision and morphological plasticity in the heterogeneous pattern, which agrees with the trend of root N concentration being higher in N enriched patches. The precise placement of fine roots promoted root N uptake. Our results about root N concentration in larch subjected to the heterogeneous pattern coincide with those of *Podocarpus macrophyllus*, *T*. *cuspidata* seedlings [11], *Ailanthus altissima* [53], and some other tree species [20, 37]. However, the increase in root N concentration did not evoke the same responses in physiological plasticity and utilization in birch seedlings. Therefore, N uptake efficiency was not modified by the heterogenous nutrient pattern in birch seedlings which resulted in the null response of N utilization. Physiological plasticity and N utilization also showed no response to the heterogeneous pattern in our larch seedlings. This is reasonable because physiological plasticity was considered to be a more expensive means to exploit nutrient enriched patches than new root construction [54]. Lack of physiological plasticity limited N use by photosynthetic organs to produce dry mass.

An improved water condition can promote N utilization both in birch and larch seedlings. The promotion of N utilization in larch was also reported by Proll et al. [55]. Larch roots can efficiently absorb N by enhancing morphological and physiological plasticity although foraging precision was not responsive to water supply [56]. Our larch seedlings also showed an increase of root N concentration with patch nutritional level, which indicated a trend of physiological plasticity of N uptake along the nutritional gradient of patches. Although we cannot find direct reference to support that birch seedlings can also obtain higher N utilization in well-watered conditions, our birch seedlings should share the same mechanism as larch because they are both sensitive to water deficit and usually dwell in the same community [34–36].

### Limit of this study

Our study has three limits. Firstly, our nutritional levels are fewer than the real conditions that birch and larch may face. More levels of patchy nutrient availabilities may result in more kinds of root foraging behavior responses. Secondly, the set of drought events in our study could be closer to the real situation if seedlings were cultured in an ambient environment instead of all-controlled chambers. Thirdly, we did not assess plasticity to the highest accuracy because we quantified total N concentration. The use of N isotope technique will greatly improve the accuracy of N uptake assessment and may lead to a different result of N utilization.

## Conclusions

Both birch and larch seedlings had common and positive responses of shoot growth to a better condition of water supply and root morphology at higher levels of patchy nutrient availability. However, the two species showed varied strategies of root foraging behavior. Birch seedlings were apt to show a better ability to forage N in higher precision and fine root morphological plasticity when exposed to the heterogeneous nutrient pattern. However, birch seedlings cannot efficiently seize N for uptake when water condition was improved. In contrast, larch seedlings did not have distinct fine root foraging precision and morphological plasticity in response to patchy N supply, but they did have an efficient root N uptake. Therefore, birch is a better dweller for acclimating to heterogeneous soil conditions and larch has a higher ability to seize N when water supply is improved.

## Supporting information

S1 Table Test for normality of standardized residuals for variables and data-transformation method for abnormal raw-data that were analyzed by pot substrate pattern or half-pot patch nutrient availability for *Betula Platyphylla* and *Larix olgensis* seedlings. (DOCX)

S1 Data (XLSX)
